# Adverse Drug Reactions in the Pediatric Population: Findings From the Adverse Drug Reaction Monitoring Center of a Teaching Hospital in Odisha (2015-2020)

**DOI:** 10.7759/cureus.19424

**Published:** 2021-11-09

**Authors:** Ratikanta Tripathy, Swarnalata Das, Palash Das, Nirmal K Mohakud, Mangalacharan Das

**Affiliations:** 1 Pharmacology, Kalinga Institute of Medical Sciences, Bhubaneswar, IND; 2 Pediatrics, Kalinga Institute of Medical Sciences, Bhubaneswar, IND; 3 Pediatric Medicine, Kalinga Institute of Medical Sciences, Bhubaneswar, IND

**Keywords:** adr monitoring centre, who-umc scale, causality assessment, children, adr

## Abstract

Background and objective

The incidence of adverse drug reactions (ADRs) in hospitalized children varies from 0.6-16.8%. There is a lack of uniformity and an absence of quality reporting with respect to the collection of data on ADRs worldwide, resulting in a scarcity of data regarding ADRs in children. In light of this, we aimed to analyze various factors related to ADRs in the pediatric population in the ADR Monitoring Center (AMC) of a teaching hospital in Odisha, India.

Methods

This was a record-based study conducted by the department of pharmacology in collaboration with the department of pediatrics. Detailed information regarding all ADR cases in children (<14 years of age) was collected in a format designed by the Indian Pharmacopoeia Commission (IPC). A total of 105 ADRs reported during a five-year period (2015-20) were subjected to analysis.

Results

The largest number of ADRs were reported in the age group zero to five years (41%). Males were affected more compared to females (1.7:1). Cutaneous ADRs were the most common type (86.5%) followed by the involvement of the gastrointestinal system (10%); 21% of cases were serious in nature, i.e., they required either hospitalization or led to a prolonged hospital stay. Antibiotics were the major drug category involved in causing drug reactions (66%) and among them, ceftriaxone (24.6%) was the most common causative agent.

Conclusions

One-fifth of the pediatric cases of ADRs were serious in nature. The most common causative agent was antibiotics, especially beta-lactams. There is an urgent need to raise awareness among healthcare professionals by conducting training programs to encourage the spontaneous reporting of ADRs, which will help to ensure drug safety in the pediatric population.

## Introduction

The World Health Organization (WHO) defines adverse drug reactions (ADRs) as unwanted reactions in humans caused by a drug on a therapeutic dose for the diagnosis, prophylaxis, or management of diseases [1]. ADRs are commonly encountered in children. The incidence of ADRs in hospitalized children ranges from 0.6-16.8% [2,3]. This is attributed to the differences in the pharmacodynamics of drugs, different body compositions, and qualitative and quantitative difference between childhood and adult diseases. Clinical trials on ADRs in this age group have been scarce, and hence there is a lack of robust information on the ADR profile of many drugs. Due to this, drugs are often used off-label or at inadequate or incorrect doses [4]. This further exposes children to the risk of ADRs. There is a lack of uniformity and an absence of quality reporting regarding the collection of data on ADRs worldwide. Since reporting of an ADR is not mandatory, it leads to further underreporting and inaccurate estimates of true incidences of ADRs. Higher rates of reporting have been observed from high-income countries, which contrasts with the situation in low- and middle-income countries. Under the Pharmacovigilance Program of India (PvPI), the Indian Pharmacopoeia Commission (IPC) is now the national coordination center after the launch of PvPI in 2010 [5]. The reporting of ADRs in India has been improving; however, there is much left to be desired. The reported incidence of ADRs from India is 2-3%, which is below that of many other nations [6]. Studies among the pediatric population are even fewer, and the reporting of data from various parts of the country lacks uniformity. A meta-analysis by Smyth et al. has shown that 7-98% of ADRs are either definitely or possibly avoidable. Keeping this in mind, we have undertaken this study to analyze the ADRs in pediatric patients reporting to our ADR Monitoring Center (AMC), which is functioning under PvPI. We focused on the pattern of ADRs including organ systems involved, with a special focus on the severity of the condition and drug categories involved.

## Materials and methods

This was a record-based study conducted in the departments of pharmacology and pediatrics at the Kalinga Institute of Medical Sciences (KIMS) in Bhubaneswar, Odisha. It is an approved AMC under PvPI since 2015. This study was approved by the Institutional Ethics Committee (IEC) at KIMS (Ref no. KIIT/KIMS/IEC/654/2021). Children aged 0-14 years attending as either outpatients or those admitted as inpatients, out of a total of 1,295,75 and 133,13 patients respectively, over five years with any suspected drug reactions, or hospitalized patients at KIMS developing a reaction to ongoing therapy administered at normal doses were included in this study.

Data collection

The information regarding ADR cases was entered into a format designed by the IPC [7]. The demographic profile (name, age, gender), details of drug reactions (chief complaints with duration, onset date, history of similar illness in the past, recovery of spontaneous nature/with treatment, seriousness), drug details (name and duration of intake of each drug, dose, and route of administration, date of intake and stoppage, indication for medication), and any related abnormal laboratory values observed were noted.

Causality and seriousness assessment of ADRs

We assessed the causality by using the WHO-Uppsala Monitoring Centre (WHO-UMC) scale and the seriousness by the WHO criteria [8,9]. For the causality assessment, information such as the temporal relationship between drug intake and the occurrence of reactions, exclusion of other causes, response to drug withdrawal (dechallenge), or rechallenge in cases of a previous history of reaction due to the same drug were collected. Based on this information, each reaction was classified into a causality category in the WHO-UMC scale: probable/possible/certain. Criteria for an ADR to be considered serious were as follows: death or life-threatening conditions among patients, or patients requiring hospitalization or suffering any permanent damage.

## Results

Out of 105 children, the largest number of ADRs were reported in the age group of zero to five years (41%). The ADR cases in the age group of 6-10 years and 11-14 years were 30.5% and 28.5% respectively (Figure 1).

**Figure 1:** Age group distribution among children with ADRs ADRs: adverse drug reactions

Males were affected more compared to females (1.7:1).

Among all the reported cases, cutaneous ADRs were the most common type (86.5%) followed by the involvement of the gastrointestinal system (10%) (Figure 2).

**Figure 2:** Involvement of different organ systems in ADRs in children ADRs: adverse drug reactions

Among ADRs affecting cutaneous systems, 48.4% of cases presented as rashes, and 29.7% cases were maculopapular reactions. Out of 105 reported ADRs, 21% of cases were serious in nature, i.e., they required either hospitalization or led to prolongation of hospital stay; 79% of cases were non-serious in nature. Three cases presented as Stevens-Johnson syndrome (SJS) were attributed to mefenamic acid, faropenem, ibuprofen, and ceftriaxone. Other serious cases observed were acute generalized exanthematous pustulosis, dapsone hypersensitivity syndrome, maculopapular drug reaction, dystonia, drug reaction with eosinophilia and systemic symptoms, red man syndrome, dystonia, hepatitis, impaired vision (due to ethambutol), bullous fixed drug eruption, and angioedema.

Antibiotics were found to be the major drug category involved in causing drug reactions (66%) followed by non-steroidal anti-inflammatory drugs (NSAIDs) (10%). It was found that a combination of antibiotics and NSAIDs was causing the reaction in 12% of cases. When a single antibiotic was taken into consideration as a causative agent for ADR, the major drug was ceftriaxone (24.6%) followed by amoxicillin (20%) (Table 1).

**Table 1:** Categories of drugs involved in ADRs in children ADRs: adverse drug reactions; NSAIDs: non-steroidal anti-inflammatory drugs; HRZE: isoniazid, rifampicin, pyrazinamide, and ethambutol respectively

Drug categories	Individual drugs (n)	Cases, n (%)
Antibiotics	Ceftriaxone (17)	69 (66%)
	Amoxicillin (14)	
	Antitubercular therapy (HRZE) (8)	
	Vancomycin (6)	
	Cefixime (3)	
	Azithromycin (2)	
	Fluoroquinolone + nitroimidazole (2)	
	Piperacillin (2)	
	Ofloxacin (2)	
	Combination of two antibiotics (6)	
	Others (7)	
NSAIDs	Paracetamol (7)	10 (9%)
	Ibuprofen (2)	
	Mefenamic acid (1)	
Anti-epileptics	Valproate (2), oxcarbazepine (2), lamotrigine (1)	5 (5%)
Antibiotic and NSAIDs	Paracetamol and antibiotics (13)	14 (13%)
	Other (1)	
Others		7 (7%)
Total		105

All the cases were subjected to causality assessment as per the WHO-UMC scale. In the majority of the cases, the drug involvement was deemed “probable” (61.5%) followed by the “possible” category in (34.5%). In four cases, the children had a history of similar reactions due to the same drug and therefore the causality link between the drug and the ADR was considered “certain”.

## Discussion

It is essential to gather as much data as possible on drug safety in the pediatric population so that the treatment of the children could be made safer. In this study, our aim was to analyze the reactions on the basis of patterns, causative drugs, and causality assessment.

Among all the reported cases, 21% of ADRs were serious in nature needing hospitalization or prolonged hospital stay, causing a financial burden to the family. Most of these cases developed during hospitalizations. ADRs in children are a major public health issue due to the unacceptably high proportion of cases that leads to considerable morbidity and mortality. A study conducted in Mexico that analyzed ADR cases from 2014 to 2017 reported that the proportion of serious ADR cases was 81%, and 70.3% were admitted to hospital because of ADRs [10]. A meta-analysis has shown the incidence of severe ADRs to be 12.3% [11]. The majority of the ADRs might not be preventable. It is found that in the majority of serious ADRs, causality assessment has shown the drugs as possible culprits. The majority of patients in our study were found to have been prescribed multidrug therapy, and we have not done a rechallenge. Also, a genetic basis needs to be ascertained to prevent the future occurrence of severe ADRs in these patients. The non-preventability of these ADRs indicates that a rational drug therapy policy needs to be followed in the hospital setup.

Antibiotics, particularly third-generation cephalosporins, contribute immensely to the problem: ceftriaxone accounts for 24.6% of ADRs if single antibiotic use as a causative agent is taken into consideration. Out of the 17 reported cases of ceftriaxone-induced ADR, 13 patients were found to have skin reactions. A retrospective study performed in China over a period of five years has shown that among all the inpatients administered with at least one dose of cephalosporin, 0.58% developed an ADR, and ceftriaxone was the most common drug involved (15.6%) [12]. We found that another beta-lactam antibiotic, amoxicillin, was responsible for 20% of cases of ADRs where a single drug was deemed a causative agent. A study done in Greece on hospitalized pediatric patients has shown that 45% of ADRs were due to amoxicillin as reported by doctors [13]. Hence, it is apparent that antibiotic stewardship is the key to preventing one-fourth of the cases of ADRs, as it lays stress on appropriate antibiotic use, thereby preventing the emergence of resistance, as well as infection control with the help of clinical pharmacology and microbiology. Beta lactam-induced reactions were predominantly found to affect the skin. Paracetamol with an antibiotic combination was responsible for 13% of cases in the possible causality assessment of total ADRs. The reactions predominantly presented as rashes, and this finding is in line with that of Titchen et al. (2005) [14].

It is found that younger children aged <5 years (41%) are the most commonly affected group by ADRs. It might be attributed to allergic reactions being lower in the younger population due to the absence of prior sensitization. However, other studies have also found that ADRs were more common in infants and pre-school children compared to children above six years [15,16]. This might be due to the fact that a large number of children under five years of age admitted to hospitals with pneumonia and diarrhea were mostly treated with empirical antibiotics. Moreover, these cases were referred cases who might have undergone polypharmacy therapy, and in the hospital, the patients were sometimes treated by multiple consultants. There were three cases of SJS in our cohort, each due to mefenamic acid, faropenem, and a combination of ibuprofen and ceftriaxone respectively. These cases required a longer duration of hospital stay leading to an immense financial burden on parents [17,18].

All ADRs were subjected to a causality assessment based on the WHO-UMC scale. A majority (61.5%) were classified as “probable” category and this finding is similar to other studies where the ADRs with a cause assessed as definite/probable ranged between 56% and 91% [19-21]. However, in our study, all the cases were not assessed for preventability; in four cases, a history of similar reactions to the same drugs was found, which led them to be deemed as “certain/definite” in the causality assessment. These cases could have been prevented by taking a proper history of previous drug reactions. In 34.5% of cases, multiple drugs were involved in causing the reaction and they were classified under the “possible” category in the causality assessment. In their study, Priyadarshini et al. applied the Naranjo scale of causality assessment and showed that 17% of cases were in the possible category.

Limitations

The present study has its share of limitations. We were unable to assess the preventability of ADRs due to the retrospective nature of the study. There are a few ADR centers in our state including the government center, but we had no opportunity to access their data. The neonatal unit of KIMS had reported very few cases, possibly due to their lack of awareness or the hectic work schedule. This might have had an impact on the results, leading to a higher proportion of older children in our cohort. Also, we have not examined the use of off-level drugs in the pediatric and neonatal unit, as it is not a part of the AMC. Moreover, we have not classified ADRs on an immunological basis, and confirmatory tests were not done to label the patients as sensitive or not as this is a report based on the data from the ADR center. Hence, the immunological basis and genetic links need to be evaluated in a multicentric study to prevent the catastrophic effect of severe ADRs.

## Conclusions

In this study, the risk of reported ADRs was inversely proportional to the age of the patients. The major drugs involved were antibiotics and the most common organ involved was the skin; 21% of cases were serious in nature. The high prevalence of serious ADRs in children might be due to the use of off-label drugs as well as healthcare professionals reporting serious cases on a priority basis. It represents a huge concern in terms of drug safety. Hence, raising awareness of ADRs among pediatricians and caregivers is of paramount importance for implementing an active ADR monitoring system for children. To reduce the risk of ADRs in children, clinicians, nurses, and pharmacists should be aware of the higher ADR risks associated with some specific drug groups.
